# Study of the kinetic, equilibrium, and thermodynamic aspects of the removal and recovery of divalent lead heavy metal ions from industrial wastewaters contaminated by vesavin-enriched XAD-11600 amberlite resin

This article has been retracted.

**DOI:** 10.1016/j.heliyon.2023.e22761

**Published:** 2023-11-24

**Authors:** Sherzod Shukhratovich Abdullaev, F. Al-dolaimy, Ahmed Hussien Alawadi, Adnan Taan Alkhafaji, Javad Zareei, Seyyed Hossein Hosseini

**Affiliations:** a Faculty of Chemical Engineering, New Uzbekistan University, Tashkent, Uzbekistan; b Engineering school, Central Asian University, Tashkent, Uzbekistan; c Scientific and Innovation Department, Tashkent State Pedagogical University named after Nizami, Tashkent, Uzbekistan; d Al-Zahraa University for Women, Karbala, Iraq; e College of technical engineering, the Islamic University, Najaf, Iraq; f College of technical engineering, the Islamic University of Al Diwaniyah, Iraq; g College of technical engineering, the Islamic University of Babylon, Iraq; h Cardiology Department, College of Medicine, Al-Ayen University, Thi-Qar, Iraq; i Department of Biosystem Engineering, Ferdowsi University of Mashhad, Iran; j Department of Mechnical Engineering, Islamic Azad University, Kashmar branch, Kashmar, Iran

**Keywords:** *Extractant-impregnated resins*, *Pb(II) adsorption*, *Amberlite XAD-11600*, *Vesavin*, *Kinetics*, *Equilibrium*

## Abstract

In this study, we developed a unique adsorbent known as extractant-impregnated resin (EIR) by surface impregnation of XAD-11600 amberlite resin with the Vesavin ligand. This resin demonstrated exceptional selectivity for the absorption of lead (Pb^2+^) ions from aqueous solutions. The ability of EIR to remove lead from polluted water was studied as a function of experimental parameters, including the kinetics, equilibrium, and thermodynamics of the adsorption process. The experimental results provided the basis for the fitting of equilibrium adsorption isotherms with the Langmuir model, and the maximum adsorption capacity of EIR for Pb(II) ions was determined to be approximately 1662 mg/g. Kinetic and thermodynamic studies were also conducted to gain insight into the behavior of the adsorption process. It was found that the rate of penetration of lead ions into the particle was the primary factor controlling the absorption process of lead on the surface of the porous adsorbent. Additionally, the studies demonstrated that the EIR can be utilized for multiple absorption and desorption cycles.

## 1 Introduction

The accumulation of heavy metals, particularly toxic metals like lead, is a significant concern in the environment. Lead, which is a ubiquitous source of environmental pollution due to its extensive usage in various industries such as battery manufacturing, poses a serious threat to human health. Controlling lead pollution and minimizing its entry into the environment has therefore become a pressing issue [[1], [2], [3]]. An effective approach for lead extraction is to utilize the recovery process. This process not only helps to reduce the lead content in wastewater but also contributes to sustainable development. However, more efforts are required to optimize these processes for efficient lead retrieval. This study explores the potential of activated carbon as an eco-friendly and cost-effective method for lead extraction from wastewater, taking into account its potential limitations and challenges [4,5].

The removal of heavy metals from wastewater is of utmost importance as these elements pose a serious threat to the environment and human health. Absorption technology is considered one of the superior methods due to its cost-effectiveness, straightforward design, ease of use, scalability, and simplicity. Chelating ion exchange resins are highly promising tools for the removal and recovery of transition metals due to their selective absorption capability based on the functional groups they contain [[2], [3], [4], [5], [6], [7], [8], [9]]. To enhance the selectivity and performance of these resins, specific ligands can be impregnated to convert neutral resins, such as XAD resins, into selective adsorbents [[10], [11], [12], [13], [14], [15]].

Studies have shown that absorption technology is a superior water treatment method in terms of cost, simplicity of design, simplicity of application, and durability for heavy metal removal applications. Weiming et al. [16] published a study that compared various wastewater treatment technologies and concluded that membrane separation technology is a promising option for treating heavy metal-contaminated wastewater. The authors noted that membrane separation has many advantages, including high efficiency, simple design, ease of use, and cost-effectiveness.

A study on wastewater treatment methods has been conducted, which provides a comprehensive overview of the various approaches available, including absorption. The study considers the pros and cons of each method and concludes that absorption is an effective, environmentally friendly, and cost-efficient technology for treating contaminated water [17].

Advanced treatment technologies for heavy metal-contaminated wastewater suggest that different methods, including membrane filtration, electrochemical processes, and absorption, can be used. The study concludes that absorption is a promising technology due to its lower cost, ease of operation, and energy efficiency [18].

Scientists and researchers have studied the absorption of heavy metals on solids for many years [[19], [20], [21], [22], [23], [24], [25], [26], [27]]. Our current study focuses on the preparation of a highly selective and recyclable Vesavin-assisted resin by impregnating the XAD-11600 polystyrene macro porous resin with Vesavin ligands, as depicted in Fig. 1. The resulting resin beads can absorb lead ions efficiently from water, and they can be conveniently desorbed and recovered using a specific detergent solution.

**Fig. 1:** The molecular structure of Vesavin.

The solid: liquid ratio and the temperature of a system can have a significant impact on the adsorption capacity, which refers to the maximum quantity of adsorbate that can be absorbed by a material [[28], [28]a],^29^]. The solid: liquid ratio refers to the ratio of the surface area of the solid to the volume of liquid in a system, and it can play a role in determining the feasibility of adsorption [30].

Equilibrium studies on Vesavin- Enriched XAD-11600 Amberlite Resin involve analyzing the behavior of the resin when it comes into contact with a particular compound to adsorb, such as an organic solvent or an analyte. These studies entail measuring the amount of the compound that is adsorbed by the resin as a function of time or equilibrium [31,32]. The results of these studies can be used to develop mathematical models that describe the equilibrium behavior of the system, which can then be used to optimize the performance of the resin in different applications. Additionally, the results of these studies can be used to compare the performance of different resins for the same application.

Comparative studies of the kinetic, equilibrium, and thermodynamic aspects of the removal and recovery of divalent lead heavy metal ions from industrial wastewater contaminated by Vesavin-enriched XAD-11600 Amberlite Resin with other materials used as adsorbents, which are existing in the specialized literature, are valuable research topics. These studies can help evaluate the performance of the different materials and identify the most efficient and economic adsorbent for the removal of lead ions [33,34]. It can also provide insights into the mechanisms of the adsorbent-adsorbate interaction, such as ion exchange, complexation, and chelation, which can be used to optimize the performance of the adsorbent [35]. The results of such studies can also be used to assess the scalability, stability, and sustainability of the adsorbent, as well as its potential for reuse and regeneration [36]. Overall, these studies can contribute to the development of new, efficient, and sustainable methods for the removal and recovery of heavy metal ions from wastewater, reducing the risk of contamination and protecting the environment [37,38].

We focused on the detailed study of the kinetic, equilibrium, and thermodynamic aspects of the lead absorption process using Vesavin/XAD-11600 resin beads in a non-continuous system. By means of semi-empirical equations, we illustrated its potential use in various industries, including water and wastewater treatment, as well as hydrometallurgy, for the efficient removal and recovery of lead metal from contaminated water and aqueous solutions. Also the experimental work carried out for the fitting of equilibrium adsorption isotherms with the Langmuir model, and the maximum adsorption capacity of EIR for Pb(II) ions determined. Beside this, Kinetic and thermodynamic studies were conducted to gain insight into the behavior of the adsorption process.

## 2 Materials and methods

### 2.1 Preparation of solutions

A lead ion solution with a concentration of 1000 mg/L was prepared using lead nitrate manufactured by Merck, Germany. During the experiments, 250 ml Erlenmeyer flasks containing 100 ml of the solution and 50 mg of impregnated resin were used for the absorption tests. Before each experiment, the flasks were cleaned by washing them with acid and then with deionized water. The lead concentrations in the solutions were measured using a flame atomic absorption spectrometer model 6800 manufactured by Shimadzu, Japan, after passing them through a Whatman filter No. 40. In all experiments, the combination of solution and adsorbent was agitated on a reciprocating shaker at a suitable speed (rpm) for effective absorption.

Temperature control was maintained throughout the experiment to ensure consistent results. Hydrochloric acid and sodium hydroxide were used to adjust the pH of the solutions at each stage. The pH of the solution was measured using a Bell Italy pH meter (model PHS-3BW) at every step of the experiment.

### 2.2 Preparation of impregnated resin

Following established methods, Amberlite XAD-11600 resin was treated with hydrochloric acid and methanol at a ratio of 1:1 for 12 h to remove any residual monomers and organic impurities. After washing with distilled water and drying with a vacuum pump, 1 g of resin was added to 200 mL of a vesavin methanol solution containing 1 % (W/W) vesavin concentration in a round-bottom flask and stirred rapidly with a shaker for 12 h to produce resin enriched with vesavin. The stabilized resin was then filtered through a sinter glass funnel, washed with acid and finally washed with distilled water to remove any remaining acid. Approximately 15 cycles of adsorption and desorption were then performed using a 0.001 M lead solution and a 0.2 M hydrochloric acid solution to remove loosely fitting ligands on the resin surface. Finally, the resin was dried in an oven at a temperature of 50–60 °C. As shown in Fig. 2, the resulting resin has a fertility ratio of 1.01 g vesavin/1 g XAD-11600, significantly improving its potency compared to the original resin. Additionally, repeated cycles of adsorption and desorption had little impact on the resin's performance as per previously published work [39].

**Fig. 2:** Photographs taken with an electron microscope (SEM) at a magnification of 30,000, showing A) XAD-11600 resin alone and B) XAD-11600 resin impregnated with Vesavin.

For all experiments, 50 mg of fertilized resin was added to 100 ml of lead solution to ensure consistent results.

XAD-11600 resin is available in two forms (Fig. 2). XAD-11600 resin alone (Fig. 2, a), which is a resin without any additional treatment, and XAD-11600 resin impregnated with Vesavin (Fig. 2, b), which is a resin that has been treated with Vesavin, an ion-exchange resin. Vesavin is used to improve the properties of XAD-11600 resin such as its capacity for the removal of organic substances, its stability, and its resistance to degradation. Therefore, XAD-11600 resin impregnated with Vesavin is typically more effective than XAD-11600 resin alone in terms of organic substance purification.

### 2.3 Absorption tests

Determining the best conditions for metal ion removal required conducting several experiments using different pH values, contact times, and models. These experiments were necessary to determine the optimal isotherm model and the kinetics of metal ion adsorption. The experiments were performed in a discontinuous system on a shaker, and the amount of metal ions remaining in the solution after each experiment was measured by flame atomic absorption spectroscopy (FAAS) to determine the amount of adsorbate removed. This allowed for the identification of the most efficient conditions for metal ion removal.

The reaction time, the amount of lead removed was calculated by calculating the difference between the initial and final concentration. The desired metal ion removal percentage and the adsorbed ion amount were then calculated using the following equations:

(1) $$R\left(\%\right)=\frac{C_{0}-C_{e}}{C_{o}}\times 100$$

(2) $$q_{e}=\frac{\left(C_{o}-C_{e}\right)v}{m}$$

where, $C_{o}$ represents the initial concentration of the metal ion in the solution, $C_{e}$ represents the final concentration of the metal ion after exposure to the adsorbent, $q_{e}$ represents the amount of metal removed, m represents the amount of adsorbent added, and v represents the volume of the metal solution.

### 2.4 Ionic exchange

Ions are a fundamental component of matter, and therefore their movement and exchange play a critical role in many natural and synthetic materials. Resins are among the synthetic materials that exploit the ionic exchange phenomenon for various applications. Ionic exchange is the process of replacing one ion in a resin with another ion from a solution. This process is important in resin technology because it enables resins to adsorb various ions from different sources.

The ionic exchange quality of resins is essential in several fields, including water treatment, food processing, and chemistry. In water treatment, resins are used to remove pollutants from water sources by adsorbing the pollutants through ionic exchange. Similarly, in food processing, resins are used to remove color, preservatives, and other substances from food by adsorbing them through ionic exchange. In chemistry, resins are used to purify compounds by adsorbing impurities through ionic exchange.

In conclusion, ionic exchange is a critical quality of resins, as it enables them to selectively adsorb and remove ions from various sources, making them useful for various applications in various fields.

## 3 Results and discussion

### 3.1 Optimal conditions of pH and ionic strength

In order to determine the optimal pH values for lead ion absorption, discontinuous experiments were conducted with the fertilized resin at different pH values (adjusted using soda and hydrochloric acid solutions). The resin was shaken in a 100 mL solution of lead ions with a concentration (100 mg/L) for 200 min. After the absorption process, the resin was separated from the solution, and the remaining lead concentration was measured using the flame atomic absorption spectroscopy (FAAS) method. According to the results, the optimal pH range for the four fertilized resins under study is 5.50–6.50, where the maximum recovery of lead is achieved. These findings are depicted in Fig. 3.

**Fig. 3:** Lead removal amount at different pH level.

The results from our study suggest that the concentration of H^+^ ions (hydronium) has an impact on the amount of lead absorbed by the fertilized resin. At lower pH values, there is increased competition between H+ and lead cations, resulting in decreased lead absorption as H+ ions are absorbed instead. As the pH increases, the concentration of H^+^ ions decreases, allowing for more lead absorption and an increase in the amount of absorption.

Despite the increased efficiency of lead absorption at certain pH levels, it is important to note that the use of caustic soda (NaOH) to adjust the pH may decrease the amount of absorption at pH values above 6.5. This is because lead ions can react with the OH- ions present in the solution, leading to the formation of an insoluble lead hydroxide (Pb(OH)2) precipitate that is not easily absorbed by the fertilized resin. Therefore, it is essential to ensure that the pH is properly adjusted and maintained throughout the absorption process to maximize lead removal.

(3) $$2Na\left(OH\right)+Pb^{2+}=Pb{\left(OH\right)}_{2}+2Na^{2+}$$

During subsequent tests, the pH of the samples was adjusted to 6 using hydrochloric acid and sodium hydroxide. The ionic strength of the samples was set to 0.01, and no significant decrease in the absorption of the desired cation was observed at an ionic strength of up to 0.3. However, it is worth noting that the optimal pH and ionic strength can vary based on the specific conditions of the experiment, such as the type of adsorbent material and the concentration and behavior of the cation in the solution. It is therefore essential to optimize these conditions for each experiment to achieve the maximum absorption efficiency.

### 3.2 Effect of stirring speed in discontinuous tests

The experiment was designed to find the optimal stirring speed for the absorption of lead ions with the use of an impregnated resin. A 100 ml solution containing 50 μg/l of lead was prepared with an optimal pH, and 0.05 g of impregnated resin was added. The solution was then shaken for 60 min at different stirring speeds (in rpm). After the absorption process, the resin was separated from the solution and washed with 5 ml of 0.2 M HCl solution, and the amount of recovered metal was measured using the presented method. Based on the results presented in Fig. 4, it was found that the rate of absorption decreased at lower stirring speeds and that a further increase in the rpm above 160 did not have a significant effect on the absorption speed. Consequently, it was inferred that 160 rpm was the optimum stirring speed for the absorption of lead ions using impregnated resin, as it resulted in the maximum recovery.

**Fig. 4:** Efficacy of lead ion removal at different stirring speeds at ambient temperature, optimal pH, and after a contact time of 60 min.

### 3.3 Investigating the mechanism and thermodynamics of adsorption

Adsorption isotherm modeling is a crucial physicochemical property involved in evaluating the appropriate characteristics of an adsorbent. Adsorption is generally measured as a function of the amount of absorption of a solute at a given concentration and temperature, under equilibrium conditions. Many isotherms, including Langmuir, Freundlich, and Temkin, have been utilized to model the uptake of dissolved substances on an adsorbent [[40], [41], [42]]. Thus, equilibrium studies have been performed to identify the best isotherm model that describes the lead absorption on the newly developed impregnated resin. This is why equilibrium data were fitted to various models, such as Langmuir, Freundlich, and Temkin, whose mathematical equations are as follows:

Langmuir model:

(4) $$q_{e}=\frac{q_{\max}bC_{e}}{1+bC_{e}}$$

Freundlich model:

(5) $$q_{e}=K_{F}C_{e}^{1/n}$$

And Tempkin model:

(6) $$q_{e}=\frac{RT}{b}\left(\ln\;K_{T}C_{e}\right)$$

Their linear form is as follows:

(7) $$\frac{C_{e}}{q_{e}}=\frac{C_{e}}{q_{\max}}+\frac{1}{bq_{\max}}$$

(8) $$\log\;q_{e}=\log\;K_{f}+\frac{1}{n}\log\;C_{e}$$

(9) $$q_{e}=B\;\ln\;K_{T}+B\;\ln\;C_{e}$$

In all the above equations, $C_{e}$ represents the equilibrium concentration (mmol.L-1), $q_{e}$ is the equilibrium absorption capacity (mmol.g-1), $q_{\max}$ is the maximum absorption capacity (mmol.g-1), b is a parameter related to adsorption energy (L.mmol-1), $K_{f}$ is the relative adsorption capacity (mmol1-1/n.L1/n.g-1), n is an experimental parameter proportional to the intensity of adsorption, B is the Temkin constant associated with the heat of adsorption (B = RT/b), and $K_{T}$ is the equilibrium bond constant (L.g-1), corresponding to the maximum bond energy. Fig. 5 show the fitting the combined data of lead ion adsorption with the Langmuir isotherm model

**Fig. 5:** Fitting the combined data of lead ion adsorption with the Langmuir isotherm model and Freundlich, and Temkin.

The isotherm curves were obtained based on the linear equations of the Langmuir, Freundlich, and Temkin isotherms. For this purpose, 100 mL of solutions with varying concentrations were prepared, onto which 0.05 g of activated resin was added. The solutions were stirred for 3 h to reach thermal equilibrium, and the metal ions were then removed using a 5 mL solution of 2.5 M hydrochloric acid detergent. The remaining concentration difference (C_0_ - C_e_) was used to calculate the amount of absorbed cation on the resin. The isotherm diagrams at ambient temperature (25° Celsius) were then generated by plotting the linear equations of the Langmuir, Freundlich, and Temkin isotherms, as illustrated in Fig. 5, Fig. 6, Fig. 7, respectively.

**Fig. 6:** Impact of time on the absorption process (initial concentration of 90 mg/L, pH = 0.6, and agitation and 160 rpm).

**Fig. 7:** Fitting the Experimental Results of Lead Adsorption on a New Fertilized Resin in a Non-continuous Agitated Reactor with the Pseudo-Lagrangian First-Order Kinetic Model: Initial Concentration of 90 mg/L, Ambient Temperature, and stirring speed of 160 rpm.

Linear isotherm graphs for the adsorption of lead ions on the resin impregnated with vesavin provided an indication that the process follows the Langmuir isotherm, suggesting a single-layer nature of the adsorption on the resin. Table 1 displays the calculated parameters for three models, namely the Langmuir model and two other models, for these ions. It can be seen that the Langmuir isotherm model best fits the experimental data, which indicates the uniform distribution of the binding sites for the adsorption of lead ions on the resin.

**Table 1:** Isotherm parameters calculated for lead ion.

Absorbent	Isotherm model	Value
	**Langmuir**	
	q_max_ (mg.g^−1^)	25/662
	b (L.mg^−1^)	6426/0
	R^2^	0000/1
	**Freundlich**	
VSV/XAD-11600	K_F_ (mg^1−(1/n)^.L^1/n^.g^−1^)	56/243
	N	13/4
	R^2^	7889/0
	**Tempkin**	
	B	23/85
	K_T_ (L.g^−1^)	88/28
	R^2^	9221/0

### 3.4 Investigating lead absorption kinetics

The Agitated Scale Reactor (ABRT) technique was used to obtain the desired kinetic model and conduct kinetic measurements, wherein a 250 mL flask was used as a reactor. A 100 mL portion of the concentrated lead solution with an initial concentration of 90 mg/L (90 mg/L) was prepared, and approximately 50 mg of fertilizing resin particles were then added to each of the solutions. The solution was stirred using a reciprocating shaker at a speed of 160 rpm, and the stirring time was recorded using a stopwatch at different periods. At specific time points, the shaker was stopped and the solution was swiftly filtered, desorbed, and the amount of absorbed lead was determined at various time points. The absorbed lead was then plotted as a function of time and different kinetic models were fitted to the data.

Fig. 6 presents the effect of stirring time on metal ion adsorption. It can be noted that the extent of metal ion adsorption increases with increasing stirring time. Nonetheless, both solvent and adsorbent appear to reach full equilibrium within 120 min or less. The experimental data presented in Fig. 6 were utilized for kinetic modeling, and several kinetic absorption models were applied to the data for analysis.

### 3.5 The pseudo-Lagrange first-order classical model

The pseudo-first-order reaction concept was introduced by Lagrange in 1898. It describes the rate of an absorption process using a pseudo-first-order rate equation, commonly expressed as [43].

(10) $$\log\left(q_{e}-q_{t}\right)=\log\;q_{e}-\frac{k_{1}}{2.303}t$$

In this study, q_t_ (mg.g^−1^) represents the amount of lead absorbed over time t, q_e_ (mg.g^−1^) is the absorption capacity in the equilibrium state, k_1_ (min^−1^) is the rate constant for the pseudo-first-order model, and t (min) is the time. The experimental data used in Fig. 6 were utilized to generate the Langmuir diagram, and the resulting plot, shown in Fig. 7.

To calculate the absorption rate constants (k1) and maximum absorption capacities (q_e_, cal) for lead ion uptake by EIR, the slope and origin of the log (q_e_ - q_t_) graphs against t were used in the pseudo-first-order kinetic model. As depicted in Table 2, the R^2 values for the Langmuir model indicate that the mechanism of lead ion adsorption on EIR grains does not follow a false first-order kinetic model. Additionally, the experimental equilibrium absorption capacity (q_e_, exp) values presented in Table 2 do not align with the calculated theoretical values utilizing equation (9), implying that the false first-order model is unsuited for modeling Pb adsorption on Vesuvine/XAD-11600 grains.

**Table 2:** Calculated parameters of several kinetic models obtained from fitting the experimental data of lead adsorption on impregnated resin using these models.

**Kinetic model**	**Values**
Pseudo first-order model (Lagrange model)	
k_1_ (min^−1^)	58/2 × 10^−2^
q_e,cal_ (mg.g^−1^)	73/165
R^2^	9933/0
Pseudo second-order model (Ho model)	
k_2_ (g.mg^−1^.min^−1^)	39/2 × 10^−4^
q_e,cal_ (mg.g^−1^)	08/196
R^2^	9547/0
Intra-Particle diffusion model	
k_ip_ (mg.g^−1^.min^−1/2^)	26/19
I	699/0
q_e,cal_ (mg.g^−1^)	∼07/198
R^2^	9989/0
Nice model	
k_0_ (mL.g^−1^.L^−1^)	00/74
Α	48/0
q_e,cal_ (mg.g^−1^)	∼52/197
R^2^	9986/0
**q**_**e,exp**_**(mg.g**^**−**^**^1^)**	**71/184**

### 3.6 Pseudo second order kinetic model

The Pseudo second-order kinetic model, first introduced in 2000 by Hong Kong scientist Professor Hu, was developed to investigate the kinetic attributes of divalent metal ions adsorbed onto coal particles under the assumption of chemical adsorption [33]. For this study, we incorporated the Pseudo second-order kinetic model to investigate the kinetic attributes of lead ions adsorbed onto Vesuvine/XAD-11600 grains. The equation for the Pseudo second-order kinetic model is presented below in its linear form.

(11) $$\frac{t}{q_{t}}=\frac{1}{k_{2}q_{e}^{2}}+\frac{t}{q_{e}}$$

In this study, the Pseudo second-order kinetic model was applied to assess the rate of the adsorption process. This model assumes chemical adsorption and the formation of a chemical bond between the adsorbent and adsorbed surface. The rate constant (K_2_) (g.mg^−1^.min^−1^) and the amount of adsorbed material (q_t_) (mg.g^−1^) at any time t (min) are used to determine the rate of the process. As such, the kinetic behavior of lead ion adsorption onto Vesuvine/XAD-11600 grains can be adequately explained by this model.

This research investigated lead ion adsorption on an impregnated resin surface using the Pseudo second-order kinetic model. Fig. 8 presents the linear plots of t/q_t_ versus t for the Pseudo second-order model, with data obtained at a temperature of 298 K. The rate constants (k_2_), R^2^ values, and the experimental and calculated values of q_e_-adsorption are compiled in Table 2 and Fig. 8. It is apparent from Table 2 that the R^2^ values are not particularly high. Additionally, it can be seen in Table 2 that the experimental values of equilibrium absorption capacity (q_e_, exp) are not in good concordance with the calculated theoretical values (q_e_, cal) per Equation (10). These inferences imply that the mechanism of lead ion adsorption on the new EIR particles does not adhere to the Pseudo second-order kinetic model, and therefore, the chemical interaction of the vesvin molecule with the lead cation is rapid and governs the rate-limiting step. Hence, the absorption rate must be sought elsewhere.

**Fig. 8:** Comparison of theoretical and experimental results of lead adsorption on newly impregnated resin in a non-continuous agitator reactor (at an initial concentration of 90 mg/l, ambient temperature and stirring speed of 160 rpm using pseudo second-order kinetic model).

### 3.7 Intra-Particle diffusion kinetic model

This model is frequently employed to model the absorption of a solute on a solid when pores or particles penetration is the rate-limiting factor, and its equation relates the amount of absorption to the root of time, expressed as the following equation [15].

(12) $$q_{t}=k_{id}t^{0.5}+I$$

Where k_id_ is the constant rate of penetration of lead into the impregnated resin grains, $q_{t}$ (mg/g) is the amount absorbed on the resin at time t, and I is a constant whose value conveys information about the boundary layer. The kinetic parameters of the Intra-Particle diffusion model were additionally calculated using the slope and y-intercept from the origin of the $q_{t}$ vs. t plot (Fig. 9), which are listed in Table 2.

**Fig. 9:** Comparison of theoretical and experimental results of lead adsorption on newly impregnated resin in a non-continuous agitator reactor (at an initial concentration of 90 mg/l, ambient temperature, and stirring speed of 160 rpm using the kinetic model of infiltration into the particles).

The values of the R^2^ parameter for the plots of penetration into the particles in Table 2 approximate 1, indicating that they are an outstanding representation. In addition, the calculated equilibrium concentrations (derived from the equations of the lines at different concentrations) at various times are slightly distinct from the experimental values, hinting at their appropriateness. The Pseudo second-order kinetic model is unique for modeling the sorption of lead on impregnated resin, and it was demonstrated that the penetration of lead ions into the pores of EIR grains is the rate-limiting step in the sorption process.

### 3.8 Thermodynamic study on the adsorption of lead onto vesavin-impregnated resin

To perform thermodynamic studies, the tests related to equilibrium (Section 3-3) were conducted at temperatures of 15, 35, and 45 °C using a water bath (Fig. 10). Based on the obtained values of the partition coefficient ($b_{m}$) at various temperatures, the required graph was plotted. The graph's slope and y-intercept from the origin allowed for the calculation of thermodynamic parameters for lead sorption on the new adsorbent, where ΔG° is always negative at all temperatures (Table 3), indicating that the process is thermodynamically favorable and takes place spontaneously at the working temperatures. The positive values of enthalpy signify an endothermic nature of the lead ion sorption process.

**Fig. 10:** Adsorption capacity curves for lead metal ion at 15, 25, and 45° Celsius

**Table 3:** Thermodynamic parameters in the absorption process of lead metal.

Temperature (°C)	b	ΔG°
15	535	−15.3
25	370	−14.7
45	291	−14.5

It can be seen that the absorption capacity ($q_{e})$ increases with the increase in the initial concentration ($C_{e})$ of the metal ion. Of course, this process is fast at first and the adsorbent has a greater inclination to absorb metal ions. Then with the decrease in the slope of the absorption curve, it is also reduced, and after the saturation stage, with the increase of the initial concentration, there is no significant change in the amount of absorbed metal ions. Also, the absorption capacity decreases with increasing temperature.

Table 3 shown that ΔG° is always negative at all temperatures, so that the process is thermodynamically favorable and takes place spontaneously at the working temperatures.

## 4 Conclusions

In this study, we have created a new adsorbent material called an extractant-impregnated resin (EIR) by impregnating and XAD-11600 resin surface with a Vesavin ligand. This resin possesses impressive selectivity towards the sorption of lead (Pb2+) ions from aqueous solutions. The removal of lead using EIR was thoroughly investigated with respect to experimental parameters, such as the kinetics, equilibrium, and thermodynamics of the sorption process. The results obtained demonstrated the following key findings.

- The maximum capacity of lead absorption by the Vesuvine-impregnated resin is improved and is reached at acidic to neutral pH levels ranging from approximately 5.5 to 6.5.
- The Langmuir isotherm represents the sorption data accurately, and the thermodynamic parameters indicate the suitability of the sorption process.
- The results revealed that the lead absorption process is governed by the penetration process into the particles, as confirmed by the fit of the data to the Weber and Morris equation in the kinetic studies.

## Additional information

No additional information is available for this paper.

## Data availability statement

Data will be made available on request.

## CRediT authorship contribution statement

**Sherzod Shukhratovich Abdullaev:** Conceptualization, Investigation, Project administration, Supervision, Writing – original draft, Writing – review & editing. **F. Al-dolaimy:** Writing – review & editing, Writing – original draft, Software, Resources, Investigation. **Ahmed Hussien Alawadi:** Writing – review & editing, Writing – original draft, Software, Resources, Investigation. **Adnan Taan Alkhafaji:** Writing – review & editing, Writing – original draft, Software, Resources, Investigation. **Javad Zareei:** Writing – review & editing, Writing – original draft, Visualization, Validation, Supervision, Software, Resources, Project administration, Methodology, Investigation, Funding acquisition, Formal analysis, Data curation, Conceptualization. **Seyyed Hossein Hosseini:** Writing – review & editing, Writing – original draft, Software, Resources, Investigation.

## Declaration of competing interest

The authors declare that they have no known competing financial interests or personal relationships that could have appeared to influence the work reported in this paper.
